# Deep Learning-Based Construction and Processing of Multimodal Corpus for IoT Devices in Mobile Edge Computing

**DOI:** 10.1155/2022/2241310

**Published:** 2022-08-05

**Authors:** Chu Liang, Jiajie Xu, Jie Zhao, Ying Chen, Jiwei Huang

**Affiliations:** ^1^School of Computer, Beijing Information Science and Technology University, Beijing 100101, China; ^2^Beijing Key Laboratory of Petroleum Data Mining, China University of Petroleum—Beijing, Beijing 102249, China

## Abstract

Dialogue sentiment analysis is a hot topic in the field of artificial intelligence in recent years, in which the construction of multimodal corpus is the key part of dialogue sentiment analysis. With the rapid development of the Internet of Things (IoT), it provides a new means to collect the multiparty dialogues to construct a multimodal corpus. The rapid development of Mobile Edge Computing (MEC) provides a new platform for the construction of multimodal corpus. In this paper, we construct a multimodal corpus on MEC servers to make full use of the storage space distributed at the edge of the network according to the procedure of constructing a multimodal corpus that we propose. At the same time, we build a deep learning model (sentiment analysis model) and use the constructed corpus to train the deep learning model for sentiment on MEC servers to make full use of the computing power distributed at the edge of the network. We carry out experiments based on real-world dataset collected by IoT devices, and the results validate the effectiveness of our sentiment analysis model.

## 1. Introduction

With the rapid development of the Internet of Things (IoT), the number of connected things is continuously increasing as well as their interactions [1–4]. At the same time, with the wide-ranging application of communication tools and several models, the IoT has been employed in the military services, medical sector, mobile communications, industrial fields, and so on [5–7]. According to the “Global IoT Device Data Report” released by International Data Corporation (IDC), it is predicted that by 2025, the number of global IoT devices will reach 41.6 billion, including all kinds of machines and sensors, smart homes, vehicles, wearable devices, and industrial equipment, and the amount of data generated annually will reach 79.4 ZB. It should be noted that data collected by IoT devices must be processed before they can be used [8].

The traditional centralized network cannot meet the needs of mobile users due to low storage capacity, high energy consumption, low bandwidth, and high latency [9, 10]. Mobile Cloud Computing (MCC), as the integration of cloud computing and mobile computing, provides considerable capabilities to mobile devices and provides them with the storage, computation, and energy resources provided by the centralized cloud. In recent years, mobile computing has shifted from centralized Mobile Cloud Computing to Mobile Edge Computing (MEC), driven by the vision of the IoT and 5G communications [11–14]. The primary function of MEC is to push mobile computing, network control, and storage to the edge of the network (for example, base stations and access points) so that the large amount of computing power and storage space distributed at the edge of the network can generate sufficient capacity to perform computation-intensive and delay-critical tasks on mobile devices [15–18]. Therefore, data collected by IoT devices can be processed by using MEC servers [19].

While emotional analysis has been successful for text, it is a question that has not been fully studied for data, which contain two or three modes of text, audio, and vision simultaneously. The biggest setbacks for studies in this direction are lack of a proper dataset and methodology [20, 21]. However, the development of IoT and MEC provides a new solution for the construction of multimodal corpus and training of sentimental analysis model. We can use IoT devices (such as IP cameras) to collect audio and vision data which contain the context information, transmit the collected data to the back-end through the network for processing and storage, and use the collected data to construct a multimodal corpus [22–24]. Then, extract the text features, audio features, and vision features of the corpus, build a multimodal sentimental analysis model based on the DialogueRNN model, deploy the model to the MEC server to make full use of the advantages of MEC server, and use the extracted text features, audio features, and vision features to train this deep learning model [25–27].

## 2. Relevant Corpora for Multiparty Dialogue in IoT

The construction of the different corpora has similarities in many aspects such as the data used, annotation process, and annotation specification, which has certain reference value for us to use the IoT devices to collect data for construction of corpus. At the same time, the construction of the different corpora can provide some guidance and reference for the data collected by IoT devices from daily life or from situation comedies. At present, English corpora are considered the most abundant resource. Therefore, this paper, starting from English multimodal corpora, introduces the related subtasks and corresponding corpora as well as the latest research work on the corpora through sorting out different multimodal sentimental analysis subtasks.

### 2.1. Bimodal Corpora

In 2016, Niu's team introduced a multiview sentiment analysis dataset (MVSA) including a set of image-text pairs with manual annotations collected from Twitter, which is annotated with positive, neutral, and negative sentimental labels [28]. The MVSA dataset consists of two parts. One is MVSA-Single, where each sample is annotated by an annotator and contains only one sentimental label, with a total of 4869 image-text pairs. The other part is MVSA-Multiple, where each sample is annotated by three annotators and contains three sentimental label, with a total of 19,598 image-text pairs. This dataset can be utilized as valuable benchmark for both single-view and multiview sentiment analysis.

### 2.2. Trimodal Corpora

#### 2.2.1. Interactive Emotional Dyadic Motion Capture

In 2008, Busso's team described a new corpus named the interactive emotional dyadic motion capture database (IEMOCAP) which contains approximately 12 hours of multimodal data to facilitate the investigations of understanding expressive human communication [29]. In total, the dataset consisted of 4,784 impromptu dialogues and 5,255 scripted dialogues with an average duration of 4.5 seconds. Each sentence in the dialogue is annotated with a specific emotional label, including anger, happiness, sadness, excitement, and frustration. The dataset also provides continuous attributes: activation, valence, and advantage. These two types of discrete and continuous emotional descriptors contribute to the complementary understanding of human emotional expression and emotional communication between people.

#### 2.2.2. Multimodal Opinionlevel Sentiment Intensity

In 2016, Zadeh's team introduced the first opinion-level annotated corpus of sentiment and subjectivity analysis in online videos called Multimodal Opinionlevel Sentiment Intensity dataset (MOSI) [30]. The sentiment intensity of data derived from YouTube videos of film reviews is defined from strongly negative to strongly positive with a linear scale from −3 to +3. The sentimental annotation of this dataset is not the feelings of the viewers but the sentimental tendencies of the speakers in the videos. A total of 93 videos which are randomly collected come from 89 narrators, all of whom express their opinion in English.

#### 2.2.3. CMU Multimodal Opinion Sentiment and Emotion Intensity

In 2018, Bagher Zadeh's team introduced CMU Multimodal Opinion Sentiment and Emotion Intensity (CMU-MOSEI), the largest dataset of sentiment analysis and emotion recognition at that time [31]. The data of CMU-MOSEI dataset are derived from the monologue videos of YouTube. This dataset which has both emotion annotation and sentiment annotation contains 23,453 annotated video segments from 1,000 distinct speakers and 250 topics. Each sentence is annotated for sentiment on a [-3,3] Likert scale of [−3: highly negative, −2 negative, −1 weakly negative, 0 neutral, +1 weakly positive, +2 positive, +3 highly positive]. Ekman emotions of fhappiness, sadness, anger, fear, disgust, surpriseg are annotated on a [0,3] Likert scale for presence of emotion x: [0: no evidence of x, 1: weakly x, 2: x, 3: highly x]..

#### 2.2.4. Multimodal EmotionLines Dataset

In 2018, Soujanya's team proposed the Multimodal EmotionLines Dataset (MELD) to solve the gap that there is no large-scale multimodal multiparty emotional conversational database containing more than two speakers [32]. The MELD dataset is derived from the EmotionLines dataset, which is a text-only dialogue from the classic TV series *Friends*. This dataset is a multimodal dataset encompassing audio, visual, and textual modalities, which contains about 13,000 utterances from 1,433 dialogues. Each utterance in the snippet of conversation is annotated with one of seven emotional labels, including anger, disgust, sadness, happiness, neutral, surprise, and fear. At the same time, each utterance is annotated with one of the three sentimental labels, including positive, negative, and neutral.

#### 2.2.5. CH-SIMS Dataset

In 2020, Yu's team proposed the Chinese single and multimodal sentiment analysis dataset (CH-SIMS) which is a fine-grained annotated Chinese multimodal emotion analysis dataset [33]. CH-SIMS dataset collected 60 original videos from movie clips, TV series, and various performance programs and cut them at the frame level. Finally, 2281 video clips were obtained. The annotator annotates each video clip in four modes: text, audio, silent video, and multimode. Each mode of each video clip is marked by 5 annotators, and the labels are divided into −1 (negative), 0 (neutral), or 1 (positive).

#### 2.2.6. DuVideoSenti Dataset

In 2021, Tang's team proposed a multimodal sentiment analysis dataset named baiDu Video Sentiment dataset (DuVideoSenti), which consists of 5,630 videos displayed on Baidu [34]. In this dataset, each video is manually annotated with a sentimental style label which describes the user's real feeling of a video. The sentimental style labels used to describe the visual and sentimental feelings of users after browsing the video in this dataset are listed as follows: hipsterism, fashion, warm and sweet, objective and rationality, daily, old-fashion, cute, vulgar, positive energy, negative energy, and others.

#### 2.2.7. Multimodal Sentiment Chat Translation Dataset

In 2022, Liang's team proposed a Multimodal Sentiment Chat Translation Dataset (MSCTD) containing 142,871 English-Chinese utterance pairs in 14,762 bilingual dialogues and 30,370 English-German utterance pairs in 3,079 bilingual dialogues [35]. Each utterance pair, corresponding to the visual context that reflects the current conversational scene, is annotated with one sentiment label (positive/neutral/negative).

## 3. Procedure of Multimodal Corpus Construction for IoT in MEC

In this section, we introduce a procedure for constructing multimodal corpus based on multiparty dialogues collected by IoT devices to provide an idea and method for researchers to construct multimodal corpus from multiple perspectives.

### 3.1. Annotation Scheme

A fundamental requirement of video fragments for constructing multimodal corpus is that the speaker's face and voice must appear in the same video fragment at the same time and it can remain for a certain period of time. In order to get the video fragments containing multiparty dialogues as raw data sources for our multimodal corpus construction as close to life as possible, we can use IoT devices to collect dialogue fragments from daily life or situation comedies as video fragments we need. At the same time, in order to effectively obtain the corresponding video fragments from the multiparty dialogues collected by IoT devices, there are also specific requirements for the collected target fragments:

1. The picture quality of the video should be as clear as possible.
2. The characters in the whole video should be as few as possible, and especially when the speaker speaks, the background characters in a video fragment should be as few as possible.
3. In a video fragment, when the speaker speaks, noise such as background music should be avoided as much as possible.

The corresponding video fragments obtained from the dialogue fragments collected by IoT devices that meet the above requirements are conducive to the annotators to determine the sentiment and emotion of the speaker appearing in the video, so as to improve the accuracy of annotation and the accuracy of the extracted features for all modalities including text, audio, and vision. In the procedure of corpus construction, in addition to ensuring the quality of video fragments to be annotated, the annotation scheme is also an indispensable part. As a result, it is necessary to develop an annotation scheme to ensure the smooth construction of multimodal corpus to meet the quality requirement of multimodal corpus and facilitate annotators to annotate.

#### 3.1.1. Annotation Unit

The annotation unit of corpus is a speech of a speaker in a dialogue. The principle of consistency should be followed when annotating each video fragment:

1. Only one speaker is allowed to speak in the same video fragment to be annotated and the emotion will not change greatly as appropriate during the speech.
2. The video fragment to be annotated should not be too short or too long by the same speaker.
3. The short sentences of the same speaker with the same emotion should be combined as appropriate, and the longer sentences should be properly segmented according to the principle of semantic integrity and consistency principle.
4. The video fragment to be annotated must meet the requirement that the people appearing on the screen must include the speaker.

If the video fragment does not conform to the above principle of consistency, the video fragment will be filtered immediately. In short, the combination and segmentation of annotation units should follow the principle of not combining the speeches of different speakers or scenarios, so that it is convenient for the annotators to annotate.

#### 3.1.2. Annotation Template

The annotation template designed in this paper includes the information of season, episode, dialogue, utterance number, speaker, utterance, emotion, and sentiment. If it is a video fragment obtained from the dialogue fragments collected by IoT devices from daily life, the information of season and episode may not be required. If it is a video fragment obtained from the dialogue fragments collected by IoT devices from situation comedies, the information of season indicates the season which a video fragment belongs to and the information of episode indicates the episode which a video fragment belongs to. The information of dialogue indicates the scene which a video fragment belongs to. The information of utterance number indicates the position of a video fragment in one dialogue. The speaker indicates the person who is talking in a video fragment. The information of utterance indicates the content text described by the current speaker. The information of emotion represents the external emotion of the person who is talking in a video fragment. The information of sentiment represents the internal feeling of the person who is talking in a video fragment, which needs to be judged by the context of the dialogue.

#### 3.1.3. Classification of Emotion and Sentiment

Sentimental information and emotional information are the focus of the whole annotation scheme. The division of sentimental categories and emotional categories is the cornerstone for the construction of the whole corpus. The standard of classification is to take into account the coverage of sentimental categories and emotional categories in the whole video. In order to reasonably organize the classification of sentiment and the classification of emotion, this paper refers to several multimodal corpora and summarizes the methods of their sentimental classification and emotional classification listed in Table 1.

It can be seen from Table 1 that the emotional classification of most multimodal corpora includes anger, disgust, fear, happiness, sadness, and surprise and the sentimental classification of most multimodal corpora includes positive, negative, and neutral. On the one hand, it strives to cover more annotation examples to make each annotation unit have accurate categories as far as possible. On the other hand, it controls the number of emotional and sentimental categories and the inclusion relationship between them to ensure the mutual exclusion of emotional and sentimental categories.

Considering the above factors and referring to the six basic emotion types proposed by Ekman [36], this paper divides sentiment into positive, negative, and neutral and divides emotion into anger, disgust, fear, joy, sadness, surprise, and neutral.

In real life, people do not necessarily show the corresponding emotions when expressing their internal feelings. Sometimes emotions conflict with people's internal feelings. At this time, it needs to be judged in many aspects to determine the character's real feelings. Therefore, when annotating sentimental information, it needs logical reasoning combined with the dialogue-context to accurately annotate the speaker's sentimental information. The annotation of emotional information only needs to be based on the external emotional expression presented by the speaker.

### 3.2. Data Preprocessing on MEC Server

Multiparty dialogues collected by IoT devices can be uploaded to MEC servers through network transmission to make full use of the amount of idle storage space distributed at the edge of the network. The procedure of data preprocessing is to use the video editing tool Adobe Premiere Pro on MEC servers to cut the target fragments at the frame level according to the consistency principle specified in the annotation unit section, which will be very time-consuming but accurate enough to obtain the video fragments that meet the requirements of multimodal corpus construction. If the video fragments collected by IoT devices are from daily life, the edited video fragment should be classified according to the scene to which the video fragment belongs. If the video fragments collected by IoT devices are from situation comedies, the edited video fragment should be classified according to the season attached, the episode attached, and the scene to which the video fragment belongs.

### 3.3. Annotation Specification

Annotation specification includes two parts: annotation principle and annotation process, which are used to control the whole procedure of multimodal corpus construction.

#### 3.3.1. Annotation Principle

When annotating sentiments and emotions, the annotated sentiments and emotions are the sentiments and emotions of the characters speaking in a video fragment, not the sentiments and emotions of the annotator watching this video fragment. At the same time, in a scene, the speaker's sentiment is easily affected by other characters in the scene, and the speaker's sentiment usually has a certain continuity in a scene. The speaker's sentiment in the preceding utterance and the sentiment in the latter utterance are likely to be the same or similar. Therefore, when annotating the sentiment of each speaker, the sentiment of the speaker should not be annotated according to the facial expression and the intonation of voice of the speaker but should be comprehensively judged according to the dialogue-context.

#### 3.3.2. Annotation Process and Quality Review

Group the preprocessed data according to the scene and then give each group of data to two persons, respectively, who annotate each group of data on the MEC servers according to the information contained in the annotation template. If the preprocessed data are collected by IoT devices from daily life, the information that should be included in the annotation template is dialogue, utterance number, speaker, utterance, emotion, and sentiment. If the preprocessed data are collected by IoT devices from situation comedies, the information that should be included in the annotation template is season, episode, dialogue, utterance number, speaker, utterance, emotion, and sentiment. The part with inconsistent sentimental and emotional information in the annotated content is handed over to the third person for judgment and decision. The process of annotation is shown in Figure 1.

The consistency of annotation is the key index to evaluate the construction of corpus. We can evaluate the quality of corpus by comparing the consistency of sentimental and emotional annotation between two annotators.

## 4. Deep Learning-Based Construction and Analysis of Multimodal Corpus for IoT in MEC

### 4.1. Building the Deep Learning Model Deployed on MEC

For our deep learning model, the overall deployment framework is shown in Figure 2.

We run our sentimental analysis model (SAM) and other strong algorithm models on a public dataset named IEMOCAP. According to the comparison results shown in Figure 3, we find that our sentimental analysis model is better than other strong algorithm models.

#### 4.1.1. Feature Extraction

*(1) Textual Feature*. Because the structure of the previous pretraining model is limited by the unidirectional language model (left-to-right language model pretraining or right-to-left language model pretraining), it also limits the representation ability of the model, so that it can only obtain unidirectional context information. BERT uses MLM for pretraining and uses deep bidirectional transformer components to build the whole model, so it finally generates deep bidirectional language representation that can integrate the left and the right context information, which is the reason why we use pretraining language model BERT to extract textual features [37]. Firstly, after the deep encoding of discourse level data by BERT, the vector at [CLS] position is taken as the feature representation of discourse level. Finally, the dimension of textual features is reduced by full connection to obtain 300-dimensional sentiment features of textual sentiment features.

*(2) Audio Feature*. OpenSMILE which is widely applied in automatic sentiment recognition in affective computing is an open-source toolkit for audio feature extraction and classification of speech and music signals, which is the reason why we use OpenSMILE to extract audio features. Firstly, we used the OpenSMILE tookit to obtain 384 dimensional sentiment features of audio, including prosodic feature and spectral feature, and then the audio features are normalized by the standard normalization (*Z*-score) method. The dimension of audio features is reduced by full connection to obtain 300-dimensional sentiment features of audio.

*(3) Visual Feature*. CNN with 3D convolutional kernels, which outperforms 2D CNNs through the use of large-scale video datasets, is intuitively effective because such 3D convolution can be used to directly extract spatiotemporal features from raw videos [38]. Firstly, the video fragment is segmented into equal frames, and then the face part in each frame is recognized and extracted. 3D CNN combined with multilayer convolution and pooling module is used to obtain the visual features contained in the video fragment. Finally, the dimension of visual sentiment features is reduced by full connection to obtain 300-dimensional sentiment features of audio.

#### 4.1.2. Sentiment Encoder

DialogueRNN is a neural network that keeps track of the individual party states throughout the conversation and uses this information for sentimental classification, which is capable of handling multiparty conversation [39]. The DialogueRNN model, which has an effective mechanism to model the context by tracking the individual speaker states throughout the conversation to classify sentiment, is based on the assumption that there are three major aspects relevant to the sentiment in a conversation: the speaker, the context from the preceding utterances, and the sentiment of the preceding utterances. It employs three gated recurrent units (GRUs) to model sentimental context in conversations. We can use the DialogueRNN model as the sentiment encoder, multimodal feature vectors as the input of the sentiment encoder, and sentimental features fused with context features as the output of the sentiment encoder.

#### 4.1.3. Deep Learning Model

After extracting the vectors of textual features, audio features, and visual features, we can splice vectors of two or three modes together to obtain the multimodal feature vectors of the current utterance on MEC server. The multimodal feature vectors are used as the input data of the sentiment encoder to obtain the representation of the sentimental feature integrating the context features. Finally, the output sentimental features are directly used as the input data of the full connection layer + softmax layer (sentiment classifier) to obtain the sentimental label of the current utterance.

### 4.2. Construction and Analysis of Multimodal Corpus for IoT

For the tens of thousands of dialogue fragments collected by IoT devices such as IP cameras from daily life, which can collect video and audio information at the same time, process the collected video and audio information to a certain extent, and transfer video and audio information to MEC servers over network, we need to select the dialogue fragments according to the specific requirements of the collected target fragments introduced in Section 3.1 to pick out the dialogue fragments that can be used to construct the multimodal corpus, which may take a lot of time and effort. However, we need to recognize the reality that although IoT devices can collect tens of thousands of dialogue fragments, most of these dialogue fragments can only ensure clear image quality but cannot ensure that there are as few characters as possible in the dialogue fragments and also cannot ensure that noise such as background music can be avoided as much as possible when the speaker speaks. These situations may lead us to pick out fewer useful fragments from the collected dialogue fragments that can be used to build a multimodal corpus. Even if these situations exist, the number of dialogue fragments collected by IoT devices that can be used to construct the multimodal corpus far exceeds the number of dialogue fragments collected by other means. At the same time, we can also use IoT devices to selectively collect the dialogue fragments we need from situation comedies, so that the collected dialogue fragments can have clear picture quality, and can ensure that there are fewer characters and less background noise in the dialogue than those directly collected from daily life.

#### 4.2.1. Construction of Multimodal Corpus

Since it takes too much time and energy to collect dialogue fragments for constructing the multimodal corpus using IoT devices from daily life, we can also collect dialogue fragments for constructing the multimodal corpus through IoT devices from situation comedies. Most situation comedies start with creating opposites and contradictions and end with solving contradictions and reaching reconciliation. Following the procedure of constructing a corpus introduced in Section 3, we choose the *Biography of the Naive WuLin*, which premiered in 2019, as the data source to construct the multimodal corpus. Compared with traditional Chinese situation comedies, this situation comedy has clearer picture quality, more obvious emotional characteristics, and less background noise, and few other characters speak at the same time when one character speaks. According to the information specified in the annotation template, some data of the constructed corpus are shown in Table 2. The speakers of *Biography of the Naive WuLin* are mainly Xiangyu Tong, Zhantang Bai, Furong Guo, Xiucai Lv, Dazui Li, Constable Xing, and Xiaobei Mo. Other supporting roles account for a small proportion.

#### 4.2.2. Analysis of Multimodal Corpus

This constructed multimodal corpus contains 5541 utterances, 330 dialogues, and 25 speakers. Figures 4 and 5, respectively, show the proportion of each sentimental type and each emotional type. In the distribution chart of sentimental proportion, neutral and negative are the two sentiments with the largest proportion, accounting for 39.67% and 38.78%, respectively. In the distribution chart of emotional proportion, neutral and joy are the two emotions with the largest proportion, accounting for 34.60% and 19.15%, respectively.  Figure 6 shows the speech proportion of each role in the corpus. Xiangyu Tong, Furong Guo, and Zhantang Bai speak the most frequently, accounting for 22.72%, 18.01%, and 16.96%, respectively, which is consistent with the role status in situation comedies because the protagonists speak more frequently in situation comedies. The average consistency of sentimental annotation in this constructed multimodal corpus is 68.5%, and the average consistency of sentimental annotation in this constructed multimodal corpus is 59.5%.

## 5. Results

Due to the limitation of space, this paper uses the constructed corpus to train the deep learning model for sentiment and analyzes the experimental results.

Figure 7 shows the experimental results of the fusion of text and audio modes. The accuracy of the prediction results after the fusion of the two modes of text and audio decreases to a certain extent compared with the accuracy of the prediction results of text mode.

Figure 8 shows the experimental results of the fusion of text and vision modes. The accuracy of the prediction results after the fusion of the two modes of text and vision is improved to some extent compared with that of the two modes of text and vision.

Figure 9 shows the experimental results of the fusion of audio and vision modes. Compared with the prediction results of audio and vision modes, the accuracy of the prediction results after the fusion of audio and vision modes is improved to a certain extent.

The above prediction results show that the accuracy of prediction results will decline after the features of audio mode and text mode are fused, which reflects that the features of audio mode and text mode have a certain conflict. Through the analysis, we find out the reasons for the above results: in the dialogue fragments collected by IoT devices from situation comedy *Biography of the Naive WuLin*, the speakers do not use Mandarin when speaking but use dialects from all over China. This is what we neglect when constructing the corpus. Due to the particularity of dialect pronunciation, there will be a certain conflict between the features of audio mode and text mode. Through the above experimental results, we should note that when collecting multiparty dialogues by IoT devices for constructing multimodal corpus, we should choose the multiparty dialogues in which the speaker speaks with standard accent.

## 6. Discussion

Our sentiment analysis model can be applied to the surveillance systems and can improve the effect of surveillance systems. The types of the surveillance system include but are not limited to empty nesters companion system and security system based on sentiment analysis. The surveillance system uses the camera and other IoT devices to obtain the video in real time and transmits the video to MEC servers. The servers analyze the sentiments of the characters in the video and take corresponding actions according to the analysis results.

### 6.1. Empty Nesters Companion System

The system can collect and obtain the sentiments of empty nesters through IoT devices such as camera equipment, sensors, and artificial intelligence technologies such as our sentiment analysis model, extract and classify the sentimental features, and transmit it to MEC servers for sentimental analysis. Then, computers give feedback according to the analysis results. The feedback forms include but are not limited to voice, image, or action. The system can use robots as the carrier to make empty nesters interact well with the system, reduce their loneliness, and increase their happiness in daily life.

### 6.2. Security System Based on Sentiment Analysis

In stations and airports, the security system based on sentiment analysis can collect the sentimental information of every tourist who passes through the security gate in real time. The system can automatically check out the people with high possibility of crime by analyzing his sentiment in a short period of time, so as to prevent criminal violations.

## 7. Conclusion

In this paper, we propose a procedure of constructing a multimodal corpus for multiparty dialogues collected by IoT devices. We construct a multimodal corpus on MEC servers according to the procedure using the multiparty dialogues collected by IoT devices. At the same time, we build a sentiment analysis model and train the model for sentiment on MEC server using the constructed multimodal corpus. According to the experimental results, we find that when collecting the multiparty dialogues by IoT devices used to construct the multimodal corpus, the speakers in the collected multiparty dialogues should preferably use the standard accent when speaking, which can improve the effectiveness of the constructed multimodal corpus. In future, we will try to use IoT devices to collect multiparty dialogue from daily life to build a multimodal corpus and continue to improve the details of the sentiment analysis model.

## Figures and Tables

**Figure 1:** The process of annotation.

**Figure 2:** The overall structure and deployment of the sentiment analysis model.

**Figure 3:** Comparison result.

**Figure 4:** The proportion of sentiment.

**Figure 5:** The proportion of emotion.

**Figure 6:** The proportion of speaker.

**Figure 7:** Result of text and audio bimode experiment.

**Figure 8:** Result of text and vision bimode experiment.

**Figure 9:** Result of audio and vision bimode experiment.

**Table 1:** Emotional and sentimental classification of other multimodal corpus.

Corpus name	Emotional classification	Sentimental classification	Source
MVSA	Null	Positive, negative, neutral	Twitter
Sarcasm in twitter	Null	Positive, negative	Twitter
Multi-ZOL	Emotional score of 1–10	Null	ZOL.com
IEMOCAP	Happiness, excitement, sadness, anger, fear, frustration, surprise	Null	Actor performance
MOSI	From strongly negative to strongly positive with a linear scale from −3 to +3	Null	YouTube
CMU-MOSEI	Happiness, sadness, anger, fear, disgust, surprise	Negative, weakly negative, neutral, weakly positive, positive	YouTube
MELD	Happiness, sadness, anger, fear, disgust, surprise and neutral	Positive, negative, neutral	TV series *Friends*
UR-FUNNY	Null	Humorous, non-humorous	TED

**Table 2:** Some data of the constructed corpus.

Season	Episode	Dialogue	Utterance number	Speaker	Utterance	Emotion	Sentiment
1	6	107	0	Xiucai Lv	Help!	Fear	Negative
1	6	107	1	Xiucai Lv	Take it easy. It hurts a little.	Sadness	Negative
1	6	107	2	Dazui Li	Tell me, how can it go on like this?	Sadness	Negative
1	6	107	3	Dazui Li	If I were you, I would apologize politely.	Sadness	Negative
1	6	107	4	Xiucai Lv	It is clear that she does not leave a little kindness to me, why should I admit my mistake?	Sadness	Negative
1	6	107	5	Zhantang Bai	Aren't you a man? Why are you mad at a little girl?	Disgust	Negative
1	6	107	6	Zhantang Bai	Look at your whole body. There's not a single intact part.	Disgust	Negative
1	6	107	7	Zhantang Bai	If you keep doing this, you're gonna die.	Disgust	Negative
1	6	107	8	Xiucai Lv	Perish together!	Anger	Negative
1	6	107	9	Xiucai Lv	Why say this sentence when there is nothing going on?	Anger	Negative

## Data Availability

The data used to support the findings of this study are available from the corresponding author upon request.

## References

[1] Huang J., Zhang C., Zhang J. (2020). A multi queue approach of energy efficient task scheduling for sensor hubs. *Chinese Journal of Electronics*.

[2] Hu L., Wu G., Xing Y., Wang F. (2020). Things2vec: semantic modeling in the internet of things with graph representation learning. *IEEE Internet of Things Journal*.

[3] Qi L., Wang X., Xu X., Dou W., Li S. (2021). Privacy-aware cross-platform service recommendation based on enhanced locality-sensitive hashing. *IEEE Transactions on Network Science and Engineering*.

[4] Huang J., Tong Z., Feng Z. Geographical poi recommendation for internet of things: a federated learning approach using matrix factorization. *International Journal of Communication Systems*.

[5] Alrowais F., Almasoud A. S., Marzouk R. (2022). Artificial intelligence based data offloading technique for secure mec systems. *Computers, Materials & Continua*.

[6] Qi L., Lin W., Zhang X., Dou W., Xu X., Jinjun C. (2022). A correlation graph based approach for personalized and compatible web apis recommendation in mobile app development. *IEEE Transactions on Knowledge and Data Engineering*.

[7] Shah H. A., Zhao L. (2021). Multiagent deep-reinforcement-learning-based virtual resource allocation through network function virtualization in internet of things. *IEEE Internet of Things Journal*.

[8] Chen Y., Xing H., Ma Z. (2022). Cost-efficient edge caching for noma-enabled iot services. *China Communications*.

[9] Orsini G., Bade D., Lamersdorf W. Computing at the mobile edge: designing elastic android applications for computation offloading.

[10] Xu X., Li H., Xu W., Liu Z., Yao L., Fai D. (2022). Artificial intelligence for edge service optimization in internet of vehicles: a survey. *Tsinghua Science and Technology*.

[11] Huang J., Wang M., Wu Y., Xuemin S., Ying C. (2022). Distributed offloading in overlapping areas of mobile edge computing for internet of things. *IEEE Internet of Things Journal*.

[12] Chen Y., Zhao F., Chen X., Wu Y. (2022). Efficient multi-vehicle task offloading for mobile edge computing in 6g networks. *IEEE Transactions on Vehicular Technology*.

[13] Zhang P., Li L., Niu K., Li Y., Lu G., Wang Z. (2021). An intelligent wireless transmission toward 6g. *Intelligent and Converged Networks*.

[14] Chen Y., Zhao F., Lu Y., Chen X. (2021). Dynamic task offloading for mobile edge computing with hybrid energy supply. *Tsinghua Science and Technology*.

[15] Huang J., Lv B., Wu Y., Xuemin S., Ying C. (2022). Dynamic admission control and resource allocation for mobile edge computing enabled small cell network. *IEEE Transactions on Vehicular Technology*.

[16] Li M., Cheng N., Gao J., Wang Y., Zhao L., Xuemin S. (2020). Energy-efficient uav-assisted mobile edge computing: resource allocation and trajectory optimization. *IEEE Transactions on Vehicular Technology*.

[17] Chen Y., Liu Z., Zhang Y., Wu Y., Chen X., Lian Z. (2021). Deep reinforcement learning-based dynamic resource management for mobile edge computing in industrial internet of things. *IEEE Transactions on Industrial Informatics*.

[18] Li M., Gao J., Zhao L., Shen X. (2020). Deep reinforcement learning for collaborative edge computing in vehicular networks. *IEEE Transactions on Cognitive Communications and Networking*.

[19] Chen Y., Gu W., Li K. Dynamic task offloading for internet of things in mobile edge computing via deep reinforcement learning. *International Journal of Communication Systems*.

[20] Zadeh A., Zellers R., Pincus E., Morency L.-P. (2016). Multimodal corpus of sentiment intensity and subjectivity analysis in online opinion videos. https://arxiv.org/abs/1606.06259.

[21] Gupta V. K., Gupta A., Kumar D., Sardana A. (2021). Prediction of covid-19 confirmed, death, and cured cases in India using random forest model. *Big Data Mining and Analytics*.

[22] Qi L., Hu C., Zhang X. (2021). Privacy-aware data fusion and prediction with spatial-temporal context for smart city industrial environment. *IEEE Transactions on Industrial Informatics*.

[23] Waggoner P. D., Shapiro R. Y., Frederick S., Gong M. (2021). Uncovering the online social structure surrounding covid-19. *Journal of Social Computing*.

[24] Jiang C., D’Arienzo A., Li W., Wu S., Bai Q. (2021). An operator-based approach for modeling influence diffusion in complex social networks. *Journal of Social Computing*.

[25] Xu J., Li D., Gu W., Chen Y. (2022). Uav-assisted task offloading for iot in smart buildings and environment via deep reinforcement learning. *Building and Environment*.

[26] Kumari R., Kumar S., Poonia R. C. (2021). Analysis and predictions of spread, recovery, and death caused by covid-19 in India. *Big Data Mining and Analytics*.

[27] Wang W., Lv Z., Lu X., Zhang Y., Xiao L. (2021). Distributed reinforcement learning based framework for energy-efficient uav relay against jamming. *Intelligent and Converged Networks*.

[28] Niu T., Zhu S., Pang L., El-Saddik A. (2016). Sentiment analysis on multi-view social data. *MultiMedia Modeling*.

[29] Busso C., Bulut M., Lee C.-C. (2008). Iemocap: interactive emotional dyadic motion capture database. *Language Resources and Evaluation*.

[30] Zadeh A., Zellers R., Pincus E., Morency L. (2016). Multimodal corpus of sentiment intensity and subjectivity analysis in online opinion videos. http://arxiv.org/abs/1606.06259.

[31] Bagher Zadeh A., Liang P. P, poria S., cambria E., morency L.-P Multimodal Language Analysis in the Wild: CMU-MOSEI Dataset and Interpretable Dynamic Fusion graph.

[32] Soujanya P., Hazarika D., Majumder N., Naik G., Cambria E., Mihalcea R. (2018). A multimodal multi-party dataset for emotion recognition in conversations. https://arxiv.org/abs/1810.02508.

[33] Yu W., Xu H., Meng F., Zhu Y., Ma Y. A Chinese multimodal sentiment analysis dataset with fine-grained annotation of modality.

[34] Tang H., Liu H., Xiao X., Wu H. (2021). A multimodal sentiment dataset for video recommendation. https://arxiv.org/abs/2109.08333.

[35] Liang Y., Meng F., Xu J., Chen Y., Zhou J. (2022). Msctd: A multimodal sentiment chat translation dataset. https://arxiv.org/abs/2202.13645.

[36] Ekman P. (1993). Facial expression and emotion. *American Psychologist*.

[37] Devlin J., Chang M., Lee K., Toutanova K. (2018). BERT: pre-training of deep bidirectional transformers for language understanding. http://arxiv.org/abs/1810.04805.

[38] Hara K., Kataoka H., Satoh Y. (2017). Can spatiotemporal 3d cnns retrace the history of 2d cnns and imagenet?. http://arxiv.org/abs/1711.09577.

[39] Majumder N., Poria S., Hazarika D., Mihalcea R., Gelbukh A. F., Cambria E. (2018). Dialoguernn: An attentive RNN for emotion detection in conversations. http://arxiv.org/abs/1811.00405.

